# Evaluation of 3D-CEUS in the Recurrence of Liver Cancer after Radiofrequency Ablation

**DOI:** 10.1155/2021/3123553

**Published:** 2021-12-20

**Authors:** Lianjie Bai, Xinping Wang, Shenglong Shi, Jian Gao, Xing Li, Ying Wang, Maitao Jiang, Chunlei Zheng, Huilin Liu

**Affiliations:** ^1^Department of Ultrasound, The Second Hospital Affiliated with Qiqihar Medical University, Qiqihar 161000, Heilongjiang, China; ^2^Department of Neurology, The Third Hospital Affiliated with Qiqihar Medical University, Qiqihar 161000, Heilongjiang, China; ^3^Department of Ultrasound, Infectious Diseases Hospital, Qiqihar 161000, Heilongjiang, China; ^4^Department of Ultrasound, The First Hospital Affiliated with Harbin Medical University, Qiqihar 150001, Heilongjiang, China; ^5^Department of Oncology Surgery, The Second Hospital Affiliated with Qiqihar Medical University, Qiqihar 161000, Heilongjiang, China

## Abstract

**Background:**

Radiofrequency ablation (RFA) has the similar curative effects to surgery, but RFA will lead to higher postoperative local recurrence rate. 3D-CEUS is a minimally invasive examination method, which is used to analyze the sensitivity to postoperative recurrence in this study.

**Methods:**

The clinical data of 60 patients with liver cancer admitted to our hospital (February 2018-February 2020) were retrospectively analyzed. All patients were treated with RFA and were followed up with 3D-CEUS, MRI, and enhanced CT examination after surgery. The ROC curve was used to analyze the differences of different examination methods in judging postoperative recurrence.

**Results:**

For the 60 patients, 52 patients (86.7%) had a single lesion and 8 patients (13.3%) had multiple lesions, with a total of 72 lesions. After RFA, 56 lesions (77.8%) were completely inactivated and 16 lesions (22.2%) remained. Totally inactivated lesions were detected as follows: 51 (91.1%) by 3D-CEUS, 42 (75.0%) by MRI, and 50 (89.3%) by enhanced CT. During a 2-year follow-up, a total of 26 recurrent lesions were detected, 24 (92.3%) by 3D-CEUS, 12 (46.2%) by MRI, and 25 (96.2%) by enhanced CT, indicating that the sensitivity of 3D-CEUS and enhanced CT was obviously higher than that of MRI (*P* < 0.001), without conspicuous difference between sensitivity of 3D-CEUS and enhanced CT (*P* > 0.05).

**Conclusion:**

As a new imaging examination method based on artificial intelligence, 3D-CEUS has a high sensitivity in patients with liver cancer who underwent RFA, which can effectively judge the recurrence after surgery and should be widely used in practice.

## 1. Introduction

Liver cancer (liver malignant tumor) mainly includes primary and secondary types, among which primary liver cancer originates from epithelial or mesenchymal tissue of liver, while secondary liver cancer is caused by invasion of other malignant tumors to liver. With the total incidence as fifth in all malignant tumors and the number of death of more than 500 thousand each year, the disease is one of the most leading causes of cancer-related death [1–3]. At present, surgery is still an important way to treat liver cancer. However, multicentricity, hepatitis, cirrhosis, and other factors pause limitation in surgery. In addition, due to the hidden onset of the disease, some patients miss the best opportunity for surgery; therefore, the treatment effect is not so satisfactory [4, 5]. With the continuous improvement of minimally invasive medical technology, transcatheter arterial chemoembolization (TACE), radiofrequency ablation (RFA), and other treatment methods have gradually become the conventional treatment of liver cancer. RFA is physical ablation treatment method, which is minimally invasive and repeatable, and can improve the safety of liver cancer treatment [6, 7]. According to some studies, the curative effect of RFA is close to that of surgery, but RFA has the defect of 3-D leakage. Therefore, some lesions cannot be completely inactivated, with the local recurrence rate after surgery of 12.3% above [8], and the recurrence rate of larger lesions is higher, with the recurrence rate of 50.0% in patients with metastatic liver cancer [9], which results in poor prognosis. Therefore, imaging examination can follow up patients treated with radiofrequency ablation, evaluate the lesion inactivation rate, and closely monitor their recurrence, which is conducive to long-term treatment effect. Previously, enhanced CT was regarded as the reliable standard for evaluating the prognosis of patients with liver cancer, but some patients were allergic to the contrast agent [10]. Compared with the above, contrast agent used in 3D-CEUS is safer. Yang et al. found that this examination method can improve the display effect of microvessels and low-speed blood flow and then reflect the perfusion of lesions [11]. The study of Tong et al. suggested that 3D-CEUS, based on artificial intelligence, was more objective, which could improve the detection rate of recurrent lesions and could help to assess the prognosis for patients and early evaluate adverse outcomes [12]. In general, 3D-CEUS is of great significance in postoperative reexamination. However, there are few studies on the application of 3D-CEUS in the evaluation of recurrence of liver cancer after RFA. This paper will explore the practical value of 3D-CEUS, which is reported as follows.

## 2. Materials and Methods

### 2.1. Research Design

This retrospective study was conducted in the hospital (February 2018-February 2020) to explore the diagnostic value of 3D-CEUS in the recurrence of liver cancer after RFA. This was a double-blind study, neither the participants nor the experimenters were aware of trial grouping, and the study designer was responsible for arranging and controlling the whole trial.

### 2.2. Research Subjects

The clinical data of 60 patients with liver cancer admitted to our hospital (February 2018-February 2020) were retrospectively analyzed. Inclusion criteria: (1) Patients met the diagnostic criteria formulated by the American Association for the Study of Liver Diseases and the Japan Society of Hepatology after pathological examination [13, 14]. (2) Patients received the whole treatment in the hospital, and no one died, transferred halfway, and stopped treatment. (3) Patients met the indications of RFA. (4) The number of lesions was under 3. (5) The diameter of a single lesion was less than 3 cm. (6) The Child-Pugh grade of patients was identified as grade A or B [15]. (7) Patients were over 18 years old. (8) 3D-CEUS, MRI, and enhanced CT were performed for patients after surgery. Exclusion criteria: (1) Patients could not be communicated with due to hearing impairment, language impairment, unconsciousness, and mental illness. (2) Patients withdrew halfway or died, and their treatment method was changed or follow-up was lost. (3) Patients had advanced cancer and presented with extensive metastasis. (4) Patients were complicated with vital organ damage. (5) The quality of images acquired by imaging examinations was suboptimal. (6) Patients received neoadjuvant radiotherapy or chemotherapy before.

### 2.3. Procedures

Sixty patients were included in the study. On the day that the patients agreed to participate in the study, the study group collected sociodemographic data and clinical data. After RFA, patients were followed up for 2 years, and the study group recorded their recurrence.

### 2.4. Moral Consideration

The study was in accordance with the principles of *Declaration of Helsinki* [16]. After enrollment, the research subjects were informed of the purpose, significance, content, and confidentiality of the study by the study group and signed the consent form.

### 2.5. Methods

All patients underwent RFA by using a radiofrequency ablation system with an output power of 1–90 W and a basic frequency of 4.6 MHz. The coagulation degree of the tissue and the human impedance could be adjusted during the surgery. Postoperative follow-up was performed by 3D-CEUS, MRI, and enhanced CT. The first follow-up time was 1 month after surgery, and the inactivation situation was evaluated by physicians. Recurrence situation was assessed in further follow-up, which was performed for 2 years after surgery. The comprehensive judgment of laboratory examination and pathological results could be served as the reliable standard for the evaluation.

#### 2.5.1. 3D-CEUS Examination

The Philips IU22 ultrasound instrument (NMPA certified no. 20123231593) that can perform 3D ultrasound imaging and Hitachi ARIETTA70 Diagnostic Ultrasound (NMPA (I) Certified No. 20103232661) that can perform 2D ultrasound imaging were used for the examination. Firstly, the patients were examined by conventional ultrasound to determine the largest section of the tumor and the best scanning position. Then, 2D-CEUS was performed. 25 mg of SonoVue (Bracco Imaging B.V., NMPA approval No. J20080052) was dissolved in 5 ml of 0.9% normal saline to prepare suspension, which was injected into the elbow vein of the patients. In addition, 0.9% sodium chloride injection (Shandong Hualu Pharmaceutical Co., Ltd., NMPA approval no. H20023428) was injected and the contrast results were recorded. After 2D-CEUS scanning, 3D-CEUS was used for examination, and suspension was made again. The same method was used for injection, and the patients were asked to hold their breath. The acquisition time of the contrast data was 30 s, and the data were stored after analysis.

After data acquisition, the ablation area was reconstructed by image processing software, and the threshold, transparency, rotation angle, and brightness were adjusted to improve the clarity and stereo of the image. After the reconstruction, three physicians with more than 10 years' experience read the films to evaluate the inactivation and recurrence rate of the lesions. The inactivation of the lesions indicated that no enhancement of ablation lesions in each stage and no expanding range of enhancement from the portal phase to the delayed phase were observed, and the microvascular structure of the lesions was completely eliminated. Manifestation of recurrence was irregular enhancement in the arterial phase and regression in the portal and delayed phases. Without reaching consensus by physicians, the conclusion was drawn after discussion.

#### 2.5.2. MRI Examination

Conventional MRI and dynamic-enhanced MRI were performed by Hitachi Echelon 1.5 T MRI Scanner (NMPA (I) certified no. 20043280047) and body surface coil. Cross section FSE-FS-T_2_WI and diffusion weighted imaging were used for conventional MRI, with TR 3500 ms, TE 84 ms, 5 mm of slice thickness, and 1 mm of slice gap. T_1_WI was TR 6.8 ms, TE 2.35 ms (in-phrase), TE 4.75 ms (opposed-phase) 5 mm of slice thickness, and 1 mm of slice gap. Dynamic-enhanced MRI was performed by injecting 0.15 mmol/kg of gadopentetate dimeglumine (Beijing Beilu Pharmaceutical Co., Ltd., NMPA approval no. H20013088) through elbow vein, and three phases of dynamic scanning were performed. Images of arterial phase, portal venous phase, and delayed phase were collected after injection of contrast medium.

Three physicians with more than 10 years' working experience read the films and evaluated the inactivation and recurrence rate of the lesions. The inactivation of the lesions indicated complete ablation of the lesions, smaller ablation area than that before treatment, and no manifestation of enhancement in dynamic-enhanced MRI. Manifestation of recurrence was annulus with uneven thickness, irregular enhancement in the arterial phase and regression in the portal phrase and enhancement less than normal liver parenchyma in delayed phase. Without reaching consensus by physicians, the conclusion was drawn after discussion.

#### 2.5.3. Enhanced CT Examination

Toshiba Aquilion 64 CT Scanner (NMPA (I) certified no. 20063300657) was used to perform plain scan for liver, with slice thickness and slice gap of 5–10 mm. 2 ml/kg of iohexol (Zhejiang Haichang Pharmaceutical Co., Ltd., NMPA approval no. H20093053) was injected through elbow vein for enhanced scan. Then, scanning was performed in arterial phase, portal venous phase, and delayed phase with tube voltage of 120 kV, tube current of 200 mA, slice thickness of 1 mm, and slice gap of 1 mm.

Volume wizard was used for reconstruction, with the thickness and interval of reconstruction of 1 mm. The multiplanar reconstruction (MPR) images were obtained by MPR technology. After the reconstruction, three physicians with more than 10 years' experience read the films to evaluate the inactivation and recurrence rate of the lesions. The inactivation of the lesions indicated no obvious enhancement in 3 stages. Manifestation of recurrence was irregular enhancement in the arterial phase and regression in the portal and delayed phases. Without reaching consensus by physicians, the conclusion was drawn after discussion.

### 2.6. Observation Criteria

1. General data: the general data table of patients was fulfilled by themselves, including the number of inpatients, name, gender, age, body weight, pathological type, lesion diameter, lesion number, lesion location, and Child-Pugh grade
2. Analysis of inactivated and residual lesions in follow-up: the detection rates of inactivated lesions by 3D-CEUS, MRI, and enhanced CT were calculated to compare the sensitivity
3. Analysis of recurrence rate in follow-up: the comprehensive judgment was regarded as the reliable standard, the diagnosis results of recurrence of liver cancer by 3D-CEUS, MRI, and enhanced CT were calculated, and the sensitivity was analyzed by ROC curve

### 2.7. Statistical Processing

In this study, the data were processed by SPSS20.0 and graphed by GraphPad Prism7 (GraphPad Software, San Diego, USA). Including enumeration data and measurement data, the study used *X*^2^ test and *t*-test. The differences were statistically significant at *P* < 0.05.

## 3. Results

### 3.1. Comparison of General Data of Patients

Sixty patients were enrolled in this study, including 35 males and 25 females, with the age of the 25–76 years old, an average age of (55.98 ± 5.68) years and an average body mass of (58.98 ± 2.65) kg. Among the 60 patients, 54 patients (90.0%) had primary liver cancer and 6 patients (10.0%) had metastatic liver cancer, with the diameter of the lesions of 1.2–8.7 cm and an average of (5.77 ± 0.24) cm. Among them, 52 patients (86.7%) had single lesions, 8 patients (13.3%) had multiple lesions, with a total of 72 lesions. There were 12 lesions (16.7%) in the left lateral lobe of liver, 18 lesions (25.0%) in the left medial lobe of liver 12 lesions (16.7%) in the right anterior lobe of liver and 30 lesions (41.7%) in the right posterior lobe of liver. The Child-Pugh grade of patients was identified as grade A or B, with 28 patients (46.7%) as grade A and 32 (53.3%) patients as grade B.

### 3.2. Analysis of Inactivated and Residual Lesions in Follow-Up

The follow-up results showed that, among 72 lesions of 60 patients, 56 lesions (77.8%) were completely inactivated and 16 lesions (22.2%) remained. Totally inactivated lesions were detected as 51 (91.1%) by 3D-CEUS, 42 (75.0%) by MRI, and 50 (89.3%) by enhanced CT. The sensitivity of 3D-CEUS and enhanced CT was significantly higher than that of MRI (*P* < 0.05), without conspicuous difference in sensitivity between 3D-CEUS and enhanced CT (*P* > 0.05); see Table 1.

### 3.3. Analysis of Recurrence Rate in Follow-Up

During 2-year follow-up, a total of 26 recurrent lesions were detected, 24 (92.3%) by 3D-CEUS, 12 (46.2%) by MRI, and 25 (96.2%) by enhanced CT, indicating that the sensitivity of 3D-CEUS and enhanced CT was obviously higher than that of MRI (*P* < 0.001), without conspicuous difference in sensitivity between 3D-CEUS and enhanced CT (*P* > 0.05); see Figure 1.

## 4. Discussion

Liver cancer is one of the malignant tumors with the highest mortality rate. Due to high risk of recurrence after treatment, imaging examination is often used in clinical follow-up to closely monitor the disease progression for patients [17]. In practice, the imaging examination of liver cancer in China has developed a complete system. Ultrasound, angiography, MRI, and CT are all common clinical examination methods. With less influence by the operator, enhanced CT is regarded as the reliable standard for examination of liver cancer after RFA [18]. This study showed that, by enhanced CT examination, totally inactivated lesions were detected as 50 (89.3%) and recurrent lesions were detected as 25 (96.2%), which was close to the general findings in the academic community. In the study of Löffler et al., 58 of 73 lesions in patients with liver metastases from colorectal cancer were completely inactivated detected by enhanced CT, with the sensitivity of 85.71% and Kappa value of 0.785 [19], indicating that this diagnostic method had high accuracy and clinical value. However, it is reported that some patients are allergic to contrast agents of enhanced CT, so it is very important to choose a safer and more efficient imaging examination method during follow-up.

Literature review has showed that enhanced CT has the advantage of objectivity. However, with the continuous development of relevant technology, this examination method in the follow-up for patients with liver cancer may be replaced [20]. Human cognition and vision are extremely complex. When analyzing still images and dynamic videos, radiologists first convert optical signals into electrochemical signals, which are transmitted to the cerebral cortex through neurons and then integrated into the consciousness [21]. Therefore, only after long-term training can radiologists read and diagnose, but the accuracy is still subject to human factors, and whether the diagnosis method is convenient or not is closely related to the time spent by manual analysis. After the 1950s, the Artificial Intelligence Laboratory of Massachusetts Institute of Technology initiated the course of computer vision. In the past ten years, the in-depth learning ability of artificial intelligence has been continuously improved [22]. In 2017, it was reported that artificial intelligence can learn and recognize liver cancer images based on different methods of in-depth learning. The classification and diagnosis system of liver diseases based on contrast-enhanced ultrasound (CEUS) imaging achieves the classification of liver diseases [23]. Some scholars have applied 2D-CEUS in the follow-up of liver cancer after surgery [24], while further development of 3D-CEUS makes imaging examination enter a new stage of microcirculation system diagnosis. This examination method can significantly enhance the echo signal of blood, which facilitates dynamic display of the blood perfusion of liver lesions. Moreover, unlike CT and MRI examination, the contrast agent used in 3D-CEUS will not diffuse into the intercellular space. Therefore, it can more accurately reflect the acoustic differences between liver parenchyma and lesions and provide more objective evaluation of lesions. It has been found in domestic and foreign literature that 3D-CEUS can effectively evaluate the inactivation of lesions by RFA [25]. In this study, among 72 lesions of 60 patients, 56 lesions (77.8%) were completely inactivated and 16 lesions (22.2%) remained. Totally inactivated lesions were detected as 51 (91.1%) by 3D-CEUS, 42 (75.0%) by MRI, and 50 (89.3%) by enhanced CT. It demonstrated that there was a high concordance between 3D-CEUS and enhanced CT for diagnosis after RFA.

At present, there is little research and no unified conclusion on whether 3D-CEUS and contrast-enhanced CT have similar effects in the diagnosis of recurrence. The results showed that during 2-year follow-up, a total of 26 recurrent lesions were detected, 24 (92.3%) by 3D-CEUS, 12 (46.2%) by MRI, and 25 (96.2%) by enhanced CT, indicating that the sensitivity of 3D-CEUS and enhanced CT was obviously higher than that of MRI (*P* < 0.001), without conspicuous difference in sensitivity between 3D-CEUS and enhanced CT (*P* > 0.05). Although the sensitivity of 3D-CEUS in detecting recurrence was slightly lower than that of enhanced CT, there was no significant difference. It should be noted that the results of this study are related to the small number of patient samples, and the practical application value of the two detection methods still needs to be further explored. At present, it is known that 3D-CEUS is safer and more convenient compared with enhanced CT, and this detection method has better application value for patients with RFA.

To sum up, 3D-CEUS has a high sensitivity in patients with liver cancer who underwent RFA, which can effectively judge the recurrence after surgery and should be widely used in practice.

## 5. Conclusion

As a new imaging examination method based on artificial intelligence, 3D-CEUS has a high sensitivity in patients with liver cancer who underwent RFA, which can effectively judge the recurrence after surgery. Based on the development status of 3D-CEUS, it is expected that 3D-CEUS can further improve the accuracy on the basis of artificial intelligence learning and has good future prospects. Further research should focus on the advantages of 3D-CEUS compared with enhanced CT.

## Figures and Tables

**Figure 1:** Analysis of diagnosis results of recurrence of liver cancer by 3D-CEUS, MRI, and enhanced CT. The abscissa was 1 − specificity, and the ordinate was sensitivity. Blue line was the examination results by 3D-CEUS, green line was those by MRI, gray line was those by enhanced CT, and the purple line was the reference line.

**Table 1:** Analysis of diagnosis results of inactivated and residual lesions by 3D-CEUS, MRI, and enhanced CT.

Comprehensive diagnosis	3D-CEUS		MRI		Enhanced CT		Total
	+	−	+	−	+	−	
+	51	5	42	14	50	6	56
−	2	14	6	10	2	14	16
Total	53	19	48	24	52	20	72

## Data Availability

The data used to support the findings of this study are available on reasonable request from the corresponding author.
